The article "A Data-Driven Customer Profiling Method for Offline Retailers" was published in 2022. Journal: Comput Intell Neurosci.

# A Data-Driven Customer Profiling Method for Offline Retailers

**DOI:** 10.1155/2022/8069007

**Published:** 2022-06-16

**Authors:** Huahong Zuo, Sike Yang, Hailong Wu, Wei Guo, Lina Wang, Xiao Chen, Yingqiang Su

**Affiliations:** ^1^Wuhan Chuyan Information Technology Co., Ltd., Wuhan 430050, China; ^2^Center of Information, Hubei Tobacco Monopoly Bureau, Wuhan 430000, China; ^3^College of Computer Science and Technology, Zhejiang University of Technology, Hangzhou 310023, China; ^4^The Southeast Digital Economy Development Research Institute, Quzhou 32400, Zhejiang, China; ^5^Jingzhou Tobacco Monopoly Bureau of Hubei Province, Jingzhou 434000, China

## Abstract

In order to accelerate the transformation of offline retailers and improve sales by using big data technology, this paper proposes a data-driven customer profile modeling method based on the collected historical purchase records of offline consumers. This method is mainly divided into three aspects: (1) an incremental RFM model is designed to classify the value of historical consumers and support the dynamic update of the model, which is more efficient than the traditional RFM model; (2) the commodity preference of different types of customers is analyzed by the TGI model, so as to guide the retail terminal to optimize the marketing strategy; (3) a commodity purchase behavior prediction model based on LSTM is proposed, which can predict the commodity that each customer may purchase in the future, so as to optimize the retail strategy. According to extensive experiments based on a true tobacco dataset, the incremental RFM model can save 80% more time than the traditional method, and our proposed prediction model can achieve 59.32% accuracy, which is better than other baselines.

## 1. Introduction

In recent years, with the transformation and upgrading of offline retail stores, smart point-of-sale terminals have become popular, enabling offline retail stores to collect consumers' historical purchase records. By analyzing these consumer data, offline retailers can optimize their resource allocation and increase consumer stickiness, which is helpful to attract consumers and improve their sales.

However, how to form an accurate and knowledge of consumers' consumption motivation, consumption ability, consumption preference, consumption habits, and consumption trends through the analysis of consumers' purchase behavior records is the main challenge at present. Therefore, this paper proposes a data-driven customer profile modeling method, which mainly includes coarse-grained value classification and preference analysis of customers, as well as fine-grained purchase behavior prediction.

Based on the consumers' purchase behavior collected by the POS terminals, we firstly use the RFM model [1] to evaluate the customers' value according to their consumption recency, consumption frequency, and consumption monetary. This paper also proposes an incremental optimization on the RFM model.

With the continuous generation of new consumer purchase behavior data, an efficient update strategy is designed to avoid the repeated reading of historical data and unnecessary redundant calculation, so as to speed up the update efficiency of the RFM model. At the same time, this paper introduces TGI (target group index) model [2], analyzes consumers' consumption habits according to their consumption records, and describes consumers' preferences according to their groups, which is conducive to recommending their preferred products according to people.

In addition, in order to help retail terminals achieve fine-grained precision marketing, this paper designs a purchase prediction model based on LSTM (long short term memory) [3], which is used to predict the commodity that the consumer is most likely to buy in the future based on his/her historical purchase behavior. To eliminate the preference biases between customers, the model takes the historical commodities purchased by a consumer in the last five times and the commodity most frequently in history as the model input and finally predicts the commodity that the consumer is most likely to buy in the future. Because the historical purchase behavior has a chronological relationship, this paper uses the LSTM model to model it. In addition, the model also uses the embedding layer [4] of the neural network to embed commodities and maps the original independent commodities into low-dimensional vectors, which can improve the prediction accuracy of the model.

The main contributions of this paper are as follows:

1. An incremental RFM model updating method is proposed, which can quickly update the old RFM model with the continuous accumulation of data.
2. We propose to use the TGI model to analyze the preference of customer groups rather than individuals, which is useful to alleviate individual bias.
3. A commodity purchase prediction model based on LSTM is proposed; it outperforms other baselines by 1.31% accuracy.

The organization of this paper is as follows: Section 2 mainly introduces the incremental RFM model; Section 3 mainly introduces the TGI model; Section 4 mainly introduces the commodity purchase prediction model based on LSTM; Section 5 carries out extensive experiments to verify the effectiveness of the proposed methods; related work is introduced in Section 6; finally, Section 7 summarizes the work of this paper.

## 2. Customer Classification Based on Incremental RFM Model

In this section, we will first introduce the relevant knowledge of the traditional RFM model, then propose our incremental RFM model update method, and finally help understand with a simple example.

### 2.1. Introduction of Traditional RFM Model

RFM model is usually used to evaluate customer churn tendency, loyalty, and customer value. This model depicts the customer dynamically through three indexes, recency, frequency, and monetary consumption. Recency means the time interval since the last transaction; frequency means the number of transactions in the last *n* months; monetary means the total cost in the last months.

The RFM model calculates the overall average value of the three indicators, records them as *r*_avg_, *f*_avg_, and *m*_avg_, *r*_avg_, and then marks the corresponding indicators as 0 or 1 according to the relationship between each customer's own RFM indicators and the average value, that is,

(1) $$\begin{array}{c} sr_{i}=\left\{\begin{array}{c} 1,\;r_{i}<r_{\text{avg}},\\ 0,\;r_{i}\geq r_{\text{avg}}, \end{array}\right.\\ sf_{i}=\left\{\begin{array}{c} 1,\;f_{i}>f_{\text{avg}},\\ 0,\;f_{i}\leq f_{\text{avg}}, \end{array}\right.\\ sm_{i}=\left\{\begin{array}{c} 1,\;m_{i}>m_{\text{avg}},\\ 0,\;m_{i}\leq m_{\text{avg}}. \end{array}\right. \end{array}$$

Based on the above formula, each customer can be marked with three 0/1 marks and finally can be classified into 8 types of consumers as shown in Table 1.

### 2.2. Incremental RFM

The three indicators of the RFM model are real-time; that is, the recency, frequency, and monetary of consumption will change with the passage of time and the generation of orders. At the same time, consumers' consumption habits and consumption demand are not invariable. It may change at any time due to consumers' new attempts, age growth, and other factors. The grab and prediction of consumers' consumption habits should be based on the “current situation.” Therefore, in order to obtain the latest RFM model, it is necessary to consider the newly generated consumption data based on historical consumption data. However, if we use the traditional calculation method to recalculate the RFM model for historical data and newly generated data, it will be very time-consuming, especially when the scale of historical data is very large. Therefore, in this section, we propose an incremental RFM calculation method to efficiently update the RFM model by counting relevant indicators of newly generated consumption data based on the historical RFM model.

For historical data, the RFM index of each consumer *i* is recorded as *R*_*i*_^old^, *F*_*i*_^old^, *M*_*i*_^old^. For the newly added data, the RFM index of consumer *j* is recorded as *R*_*j*_^new^, *F*_*j*_^new^, *M*_*j*_^new^. In order to update the old RFM model, we need to consider the new data. At this time, the following three situations will occur:

Case 1: the consumer *u* has purchase records in both historical data and new data:
  (2) $$\begin{array}{c} R_{u}=R_{u}^{\text{new}},\\ F_{u}=F_{u}^{\text{old}}+F_{u}^{\text{new}},\\ M_{u}=M_{u}^{\text{old}}+M_{u}^{\text{new}}. \end{array}$$
Case 2: the consumer *u* only has purchase record in the historical data, and there is no purchase record in the new data:
  (3) $$\begin{array}{c} R_{u}=R_{u}^{\text{old}}+I,\\ F_{u}=F_{u}^{\text{old}},\\ M_{u}=M_{u}^{\text{old}}, \end{array}$$
where *I* indicates the time interval of new data. If we update the RFM model every month, then *I* = 30.
Case 3: the consumer *u* only has a purchase record in the new data, but there is no purchase record in the historical data:
  (4) $$\begin{array}{c} R_{u}=R_{u}^{\text{new}},\\ F_{u}=F_{u}^{\text{new}},\\ M_{u}=M_{u}^{\text{new}}. \end{array}$$

After the RFM indicators of each consumer are updated, the average value of each indicator needs to be calculated before consumers can be classified. Suppose that the consumer set in the historical data is recorded as *U*^old^, including *N*^old^ consumers, and the average RFM values of the historical data are *R*_avg_^old^, *F*_avg_^old^, *M*_avg_^old^. Suppose that the consumers in the new data are recorded as a combination of consumers *U*^new^, including *N*^new^ consumers who have purchase behavior in the historical data, and *N*_2_^new^ consumers who have no purchase behavior in the historical data, and then they meet *N*_1_^new^ + *N*_2_^new^=*N*^new^. The average value of each index of the updated RFM model can be calculated by the following formula:

(5) $$\begin{array}{c} F_{\text{avg}}=\frac{\left(F_{\text{avg}}^{\text{old}}\times N^{\text{old}}+\sum_{j\in U^{\text{new}}}F_{j}^{\text{new}}\right)}{\left(N^{\text{old}}+N_{2}^{\text{new}}\right)},\\ M_{\text{avg}}=\frac{\left(M_{\text{avg}}^{\text{old}}\times N^{\text{old}}+\sum_{j\in U^{\text{new}}}M_{j}^{\text{new}}\right)}{\left(N^{\text{old}}+N_{2}^{\text{new}}\right)},\\ R_{\text{avg}}=\frac{\left(\sum_{i\in U^{\prime }}\left(R_{i}^{\text{old}}+30\right)+\sum_{j=1}^{N^{\text{new}}}R_{j}^{\text{new}}\right)}{\left(N^{\text{old}}+N_{2}^{\text{new}}\right)}, \end{array}$$

where *U*′=*U*^old^ − (*U*^old^∩*U*^new^) represents the consumer set with purchase records only in the historical data.

## 3. Examples

Assume that we have obtained RFM results for four consumers based on the historical data, as shown in Table 2:

The average value of each indicator can be calculated:

(6) $$\begin{array}{c} r_{\text{avg}}=\frac{1}{4}\left(33+34+36+37\right)=35,\\ f_{\text{avg}}=\frac{1}{4}\left(3+1+3+1\right)=2,\\ m_{\text{avg}}=\frac{1}{4}\left(28+27+26+59\right)=35. \end{array}$$

Then, according to the relationship between the RFM data of each consumer and the average value, calculate the scoring of each consumer in the three indicators, and *u*1 is used as an example:

(7) $$\begin{array}{c} r_{1}=33\;<\;r_{\text{avg}}=35\;\Rightarrow \;sr_{1}=0,\\ f_{1}=3>\;f_{\text{avg}}=2\;\Rightarrow \;sf_{1}=1,\\ m_{1}=28>\;f_{\text{avg}}=35\;\Rightarrow \;sm_{1}=0. \end{array}$$

Similarly, the scoring matrix of all consumers can be obtained, as shown in Table 3:

According to Table 1, the consumer classification results of the four consumers are shown in Table 4:

It is assumed that another month has passed on the basis of Table 2, and the data volume of one month has been increased, and the RFM statistics of this month are shown in Table 5:

A new consumer *U*5 is added, which has not appeared in Table 2 before. In addition, *U*2 and *U*4 are not recorded in Table 5 because they have not bought goods within this month.

According to Tables 2 and 5, it can be calculated that *N*^old^=4, *N*_2_^new^=1, *F*_avg_^old^=2, *M*_avg_^old^=35, *U*′={*u*2,  *u*4}, so according to the formula in Section 2.2,

(8) $$\begin{array}{c} F_{\text{avg}}^{\text{new}}=\frac{2*4+2+1+2}{4+1}=2.6,\\ M_{\text{avg}}^{\text{new}}=\frac{35*4+18+15+18}{4+1}=38.2,\\ R_{\text{avg}}^{\text{new}}=\frac{\left(34+30+37+30+10+2+5\right)}{4+1}=29.6. \end{array}$$

It can be seen that the incremental method does not need to traverse the historical data to obtain the historical RFM value, which saves much time.

### 3.1. Product Preference Analysis Based on TGI Index

Target group index (TGI), also known as the target group index, can reflect the strength or weakness of the target group within a specific research scope. In short, it is the preference of the target group for an object or feature compared with all members. The TGI index can be calculated by the following formula:

(9) $$\begin{array}{c} \text{TGI}=\frac{\text{Proportion of certain characteristics in the target group}}{\text{Proportion of groups with the same characteristics in the population}}\;*100\text{\%}. \end{array}$$

TGI index represents the difference of different groups on the same problem. TGI index equal to 100 indicates the average level, and an index higher than 100% indicates that such consumers pay more attention to a certain problem than the overall level. For example, assume that there are 35% of people smoke in China, and 50% of Chinese men smoke. Therefore, we can calculate that TGI = 50/35 ∗ 100% = 142%, indicating that Chinese men prefer smoking than women.

Based on the classification results of the RFM model in Section 2, we will use the TGI model to analyze the preference of different categories of customers for various goods. The general flow of analysis is shown in the Figure 1.

Firstly, we will use the RFM model to classify customers (red arrow part), then select the four goods with the highest sales volume from the historical data for analysis, and calculate the TGI index of eight types of consumers (blue arrow part). Through the TGI index, we can analyze the preferences of different types of customers, so as to provide suggestions for the replenishment of retail terminals in the future.

## 4. The Commodity Purchase Prediction Model Based on LSTM

Consumers' purchase behavior can be regarded as sequential data, and traditional machine learning can be used. However, the ability of traditional machine learning methods to capture time-series correlation characteristics is weak, while the recursive neural network (RNN) [5] in deep learning can handle time-series correlation data well. Therefore, in this section, we will use the framework of the recursive neural network to predict commodity purchase behavior.

### 4.1. Introduction of the LSTM Model

The traditional RNN model structure is shown in Figure 2. The data of each time step is composed of the input data of the current time and the data of the previous time step. Each edge of the input and output has weights, which are *W*, *U* and *V* respectively. RNN network mainly includes two important processes, forward propagation of data and backward propagation of gradients. The parameters of the model are adjusted through forward and backward propagation to optimize the network. However, the traditional RNN model will have the problem of vanishing gradient or exploding gradient [6] with the increase of time step, so someone later optimized the RNN model and proposed the long and short memory neural network (LSTM) [3].

On the basis of RNN, LSTM adds input gate, output gate, and forget gate to make the model selectively remember important data and forget unimportant data and further optimize the prediction method of RNN. The input gate determines the update of information, and the output gate determines the information output of the cell state. Through the gate structure, important information is saved, and unnecessary information is forgotten to improve the memory of long-term sequences. The calculation of each gate of LSTM is shown in equations (10)–(15). The structure of LSTM is shown in Figure 3.

(10) $$\begin{array}{c} f_{t}=\sigma \left(W.\left[h_{t-1},x_{t}\right]+b_{i}\right), \end{array}$$

(11) $$\begin{array}{c} \tilde{C_{t}}=\text{tanh}\left(W_{C}.\left[h_{t-1},x_{t}\right]+b_{i}\right), \end{array}$$

(12) $$\begin{array}{c} i_{t}=\sigma \left(W_{i}.\left[h_{t-1},x_{t}\right]+b_{c}\right), \end{array}$$

(13) $$\begin{array}{c} C_{t}=f_{t}*C_{t-1}+i_{t}*\tilde{C_{t}}, \end{array}$$

(14) $$\begin{array}{c} o_{t}=\sigma \left(W_{o}\left[h_{t-1},x_{t}\right]+b_{o}\right), \end{array}$$

(15) $$\begin{array}{c} h_{t}=o_{t}*\text{tanh}\left(C_{t}\right). \end{array}$$

### 4.2. The Prediction Model Based on LSTM

In this section, we design a commodity purchase prediction model based on LSTM, as shown in Figure 4. Firstly, it takes the commodities purchased by the consumer for the first five times as the time-series feature, which is recorded as *X*1, *X*2, *X*3, *X*4, and *X*5. It also takes the most frequently purchased commodity in history as the additional feature, which is recorded as *TzX*6. The model inputs them into the embedding layer [7] and maps each commodity into a low-dimensional vector representation. The vector representation of each commodity implies the correlation between commodities and their respective characteristics, which can help the prediction model better analyze the historical behavior of consumers.

After embedding, *X*1 to *X*5 are fed into LSTM neural network and output the final hidden layer result *P*. The hidden layer result *P* integrates the characteristics of the consumer's previous five purchase behaviors and then maps to a deeper feature space through a layer of full connection, which is recorded as *P_C*.

As an additional feature, the most frequently purchased commodity in the consumer's history has no sequential relationship with the commodities that are purchased in the last five times, so it is not processed by LSTM neural network. We input the embedding representation of *TzX*6 into a fully connected layer and map it to *P_A*, whose dimensions are the same dimension as *P_C*, written as *TZ_C*. Then, we concatenate *P_C* and *TZ_C* and fed them into two fully connected layers to produce the final prediction result *Y_predict*.

Because there are many commodities that can be predicted, the prediction task actually is a multiclassification problem. Therefore, the final model output *Y_predict* is a multidimensional vector, and the corresponding number of each dimension in the vector represents the probability that the consumer purchases the corresponding commodity. We can take the commodity represented by the one dimension with the greatest probability as the final prediction result.

Therefore, we adopt the cross-entropy loss [8] as the loss function of the model. Then, we adopt the Adam [9] gradient optimization algorithm to optimize model parameters according to the error between prediction and ground truth.

## 5. Experiments

In this section, we will use the real consumer consumption records collected by cigarette sales terminals in a prefecture level city of Hubei Province from June 9, 2019, to March 9, 2021, for experimental verification. Our experimental data is from the real purchase records generated by customers in commodity enterprises. On this basis, we preprocessed and annotated the data. Each record of data contains the customer's last five purchases, the most frequently purchased commodity and labels. Through data cleaning and preprocessing, the final data includes 371089 consumers and 51095 purchase records, including 1655 cigarette brands.

Firstly, we conduct efficiency experiments on the incremental RFM model to study the time cost in updating the RFM model in different ways and verify the effects of the incremental calculation method proposed in this paper. Secondly, we display the TGI results of the top-4 cigarette brands based on classified consumers by the RFM model. Finally, we test the accuracy of the prediction model based on LSTM and compare its accuracy with different classification models, so as to verify the prediction effect of the proposed model. At the same time, we also conducted some ablation experiments to analyze the performance differences of the model under different conditions.

In the purchase prediction experiment, we conducted a 10-fold cross validation and then calculated the average and standard deviation of the experimental results as the final performance of models.

### 5.1. RFM Efficiency Experiments

In order to compare the update efficiency of the incremental RFM model before and after optimization, based on the data of one and a half years (2019/6/9–2020/2/9), we compared the calculation time after adding new data of different *D* days, in which *D* takes 7, 14, 21, 28, 35, and 42. In order to avoid accidental errors, we run the program several times to calculate the average running time (see Figure 5).

As can be seen from Figure 5, with the increase of new data, the incremental RFM model can save about 5 seconds than the tradition RFM model, which means that our proposed method can greatly improve the efficiency of update the model (the updating model).

### 5.2. TGI Results

According to statistics, the four kinds of cigarettes with the highest sales volume in history are yellow crane tower (soft blue), Liqun (new version), Yellow Crane Tower (hard wonder), and Red Golden Dragon (soft boutique).  Figure 6 shows the TGI index of eight categories of customers.

Taking Yellow Crane Tower (soft blue) as an example, the TGI index of important value consumers is 929.925%, which is much higher than the measurement standard of 100%, which shows that important value consumers have a high preference for Yellow Crane Tower (soft blue) compared with other consumers; the TGI index of important retained consumers is only 48.125%, far lower than 100%. In proportion, few important retained consumers buy Yellow Crane Tower (soft blue).

If the four products with the highest sales volume are compared horizontally, it is not difficult to find that these four products are more popular with the four types of consumers: general maintenance consumers, important maintenance consumers, general value consumers, and important value consumers, especially the important maintenance consumers and important value consumers, while the Yellow Crane Tower (hard wonder) and Red Golden Dragon (soft Boutique) are also popular with important development consumers. In contrast, important value consumers prefer Liqun (new version), important maintenance consumers and important development consumers prefer Hongjinlong (soft boutique), and important retention consumers prefer yellow crane tower (hard spectacle).

### 5.3. Accuracy Evaluation of the Prediction Model Based on LSTM

In this section, we will compare the accuracy of the cigarette purchase prediction model based on LSTM proposed in this paper with other machine learning algorithms, including support vector machine (SVM) [10], random forest (RF) [11], decision tree (DT) [12], and XGBoost [13]. The parameters of each model are determined according to the prediction results after careful grid search.

Figure 7 shows the accuracy comparison results of the five methods, where the blue bar represents the average accuracy and the green bar represents the standard deviation of accuracy. It can be seen from the figure that the method proposed in this paper achieves the highest accuracy, reaching 59.32%. It is 1.31% better than the second-place method (XGBoost). And the standard deviation of the method proposed in this paper is lower, which shows that our method has better robustness and can better deal with data anomalies.

Secondly, in the comparison methods, we can see that the prediction algorithm based on the tree is better than SVM, probably because the prediction model based on tree can potentially describe the temporal relationship of purchase behavior according to the splitting order of tree nodes.

### 5.4. Ablation Study

In this section, we will compare the impact on the LSTM cigarette purchase prediction model by 3 key factors, which are the embedding layer in the model, and the characteristics of the most frequently purchased cigarettes in the data, and the characteristics of the previous *K* purchases.

### 5.5. Influence on Prediction Effect of the Embedding Layer

In this section, we study the impact of the embedding layer by comparing the prediction accuracy of models with and without an embedding layer (see Figure 8).

In Figure 8, the blue bar graph represents the mean value of accuracy and the green bar represents the standard deviation of accuracy. When there is an embedded layer in the model, the average accuracy rate reaches 59.32%, which is 16.77% higher than that without this layer. It can be found that the average accuracy rate is greatly improved. In addition, the standard deviation of accuracy is also reduced by 1.86% compared with that without the embedding layer, indicating that the prediction effect of the model is more stable when this layer is added. Therefore, the embedding layer is useful to improve the prediction accuracy of the model.

### 5.6. Effects of the Most Frequently Purchased Commodity

In this section, we study the impact of the most frequently purchased good by comparing the prediction accuracy of models with and without this feature, and the results are shown in Figure 9.

In Figure 9, the blue bar represents the average value of accuracy and the green bar represents the standard deviation of accuracy. It can be seen from the figure that the accuracy with *TzX*6 in the feature reaches 59.32%, which is 7.62% higher than that without *TzX*6. In addition, the standard deviation is reduced by 3.4%, which makes the prediction effect of the model more accurate and more stable.

### 5.7. Effects of Previous *K* Purchase Records

In this section, we compare the impact on the prediction effect of consumers' recent *K* different purchase behaviors.

Figure 10(a) compares the average accuracy of five different *K* consumption records. It can be seen from the figure that the prediction accuracy first decreases and then increases with the increase of the *K* value. When *K* is 5, the accuracy of the model is more than 0.92% higher than the average accuracy when *K* is 2, 3, and 4. It is interesting that when we only consider the latest purchase record, the model achieves the best performance. It indicates that the consumer's purchase behavior is most related to his/her latest purchase behavior and his/her long-term behavior.

In Figure 10(b), it compares the standard deviation of accurate values of five different *K* values. It can be seen that, among the last four *K* values, the standard deviation of five consumption records is the smallest, reaching 9.32%, indicating that the prediction effect is the best and most stable when *K* = 5. Similarly, when *K* = 1, although the standard deviation is relatively small, the randomness of the customer's latest record is relatively large, which cannot explain the customer's long-term consumption preference and consumption habits. Therefore, considering the prediction effect and significance of each *K* value, five is a better choice than one.

## 6. Related Work

The main work of this paper is to carry out customer profiling work, so we first investigate the work related to the customer profiling. Besides, we improve the traditional RFM model and classify customers by the incremental RFM model. And we solve the commodity purchase predictions problem. Therefore, we further investigate the related work into the RFM model and commodity purchase predictions.

 
*Customer profiling*: In the trend of a big data environment, customer profiling is used more and more in online shopping and offline retail. In 2016, Li et al. [14] used the *K*-means algorithm to divide different cigarette attributes and customer attributes and proposed the retailer with the format of the grocery store, the market type of city, the regional type of school district, and the business scale of medium scale. Customers recommend flue-cured cigarettes. In the product recommendation problem in 2019, Zhou et al. [15] proposed a multimodel stacking ensemble (MMSE) algorithm for the personalized product recommendation problem, which is mainly divided into data analysis and model construction. In the data analysis section, Zhou et al. proposed a feature model containing six feature clusters. They designed a sampling algorithm to balance the ratio of positive and negative samples through *k*-means clustering and undersampling. In the construction of customer profile in the new retail environment proposed by Wang [16], the author takes the customer of offline stores and online stores on the “Tesco on Campus” platform as the research object, based on the essential attribute characteristics of customers, consumer behavior characteristics. There are three dimensions of time and space features, and the data is analyzed by clustering, and the RFM model is constructed using the time and space feature dimensions. Different from the above work, the incremental RFM model is first proposed, and then it used to classify customers. And we solve the commodity purchase predictions problem. This approach helps us construct customer profiling from multiple perspectives.
 
*RFM model*: Different researchers have improved the traditional RFM model to varying degrees. For example, Ye [9] designed the online consumer value RFM from three dimensions. Wei [17] proposed adding customer demographic characteristics to the RFP model by combining qualitative and quantitative analysis, breaking the traditional collaborative filtering algorithm based on the RFM model. Anitha and Patil [18] combined the RFM model and *K*-means clustering method to classify customers. Khajvand et al. [19] extended the RFM model and introduced a new counting parameter to classify customers. You et al. [20] used the RFM and decision-making models for precision marketing. Different from the above work, starting from the update efficiency of the RFM model, this paper proposes an incremental RFM calculation method. Based on historical RFM model, it counts relevant indicators of newly generated consumption data and quickly updates the RFM model.
 
*Commodity purchase predictions*: Commodity purchase predictions mostly use machine learning and deep learning methods in purchase behavior prediction. With the gradual deepening of research, some multistage hybrid models have been derived from the single initial model. Ge et al. [21] established an overall customer behavior feature model by constructing customer behavior feature engineering and designed a customer purchase behavior prediction method based on deep forest, which achieved an efficient behavior prediction training effect. XGBoost algorithm is based on Bagging strategy in commodity purchase prediction proposed by Dongqing and Chengji [22]. After that, researchers gradually realized that commodity purchase prediction is essentially a time-series prediction problem. Therefore, some e-commerce commodity prediction problems use related single models or multistage hybrid models based on deep learning and neural network models. For example, Xuyang and Fengjing [23] proposed a prediction model based on the combination of LSTM and random forest. In commodity purchase predictions, Yin et al. [24] designed a customer profiling based on TF-IDF customer cigarette preference prediction algorithm model based on a tobacco company, combining customer portraits and customer preference prediction. The character data author uses TF-IDF to analyze and predict the customer's emotional tendency towards commodity. The text-based data predicts the customer's preference value for cigarettes by calculating the similarity of the data. Due to the lack of mature customer preference and commodity purchase predictions models in cigarette companies, the TF-IDF prediction model only considers the purchase frequency of customers and does not consider the time-series nature of commodity purchase predictions. Different from the above work, based on the LSTM model, this paper uses six fine-grained features to make predictions, and the fine-grained data include the last five purchases of consumers and the most frequently purchased goods. Commodity purchase predictions consider the customer's commodity purchase frequency and the timing of the customer's purchase behavior and can make dynamic and accurate predictions based on changes in customer behavior in recent times.

## 7. Conclusions

This paper proposes a consumer profiling method from three aspects by using the historical purchase records of consumers collected by retail terminals. Firstly, an incremental RFM model is designed to classify customers' value and judge whether customers are valuable and loyal. The incremental RFM model can achieve model update in a shorter time than the traditional method. Then, the TGI model is used to analyze the preference of classified customers. Although we only analyze the top four well-sell cigarette brands in experiments, it can be easily extended to other goods of interest. Finally, we propose a commodity purchase prediction model based on LSTM to predict which commodity will be bought by each customer in the future. We take the customer's last five purchase records and the most frequently purchased commodity in history as the input features and adopt semantic embedding and LSTM model to predict the final results. Through experiments on real cigarette purchase data, it is verified that the model can achieve the best prediction accuracy, reaching 59.32%.

In future work, we will continue to optimize the commodity prediction model, hoping to mine the patterns of consumer interest changes and improve the prediction accuracy of the model.

## Figures and Tables

**Figure 1:** TGI analysis process.

**Figure 2:** RNN model.

**Figure 3:** LSTM model.

**Figure 4:** The architecture of the prediction model.

**Figure 5:** Comparison of RFM model efficiency.

**Figure 6:** TGI index of TOP-4 well-sell cigarettes by different categories of customers. (a) Yellow crane tower (soft blue). (b) Liqun (new version). (c) Yellow crane tower (hard wonder). (d) Red golden dragon (soft boutique).

**Figure 7:** Comparison of model evaluation results.

**Figure 8:** Comparison of effect with and without embedding layer.

**Figure 9:** Comparison of effect with and without *TzX*6 feature.

**Figure 10:** Comparison of different *K* consumption records. (a) Average accuracy. (b) Average standard deviation.

**Table 1:** Consumer classification of RFM model.

Consumer classification	Type	Recency	Frequency	Monetary
Important value consumers	1	1	1	1
Important development consumers	2	1	0	1
Important maintain consumers	3	0	1	1
Important retain consumers	4	0	0	1
General value consumers	5	1	1	0
General development consumers	6	1	0	0
General maintain consumers	7	0	1	0
General retain consumers	8	0	0	0

**Table 2:** Consumer RFM table based on historical data statistics.

Consumer	Recency	Frequency	Monetary
*u*1	33	3	28
*u*2	34	1	27
*u*3	36	3	26
*u*4	37	1	59

**Table 3:** Consumer RFM scoring table based on historical data statistics.

Consumer	Recency	Frequency	Monetary
*u*1	0	1	0
*u*2	0	0	0
*u*3	1	0	0
*u*4	1	1	1

**Table 4:** RFM results based on historical data statistics.

Consumer	Classification
*u*1	General maintain
*u*2	General retain
*u*3	General develop
*u*4	Important value

**Table 5:** RFM results in the latest month.

Consumer	Recency	Frequency	Monetary
*u*1	10	2	18
*u*3	2	1	15
*u*5	5	2	18

## Data Availability

The dataset used were collected from the tobacco monopoly bureau and are not publicly accessible.
